# Fault Diagnosis of Wind Turbine Based on Convolution Neural Network Algorithm

**DOI:** 10.1155/2022/8355417

**Published:** 2022-07-16

**Authors:** Wei Xiao, Zi Ye, Siyu Wang

**Affiliations:** ^1^School of Electrical and Information Engineering, Anhui University of Science and Technology, Huainan 232001, China; ^2^Guohua Energy Investment Co., Ltd., Beijing 100007, China; ^3^State Grid General Aviation Co., Ltd., Beijing 102209, China; ^4^Institute of Modern Supply Chain, Chinese Academy of International Trade and Economic Cooperation, Beijing 100013, China

## Abstract

Relying on expert diagnosis, it solves the problem of fan failure efficiency and meets the needs of automatic inspection and intelligent operation monitoring of fans. In order to make up for the deficiency of intelligent diagnosis of bearing fault based on vibration signal detection, signal transformation, and convolution neural network identification and improve the ability of intelligent diagnosis, this study designs a deep convolution neural network model and diagnosis algorithm with three pairs of convolution pooling layers and two full connection layers. The experimental verification of the proposed method is carried out based on the public data set, and the effects of three different signal transformation methods based on vibration signal through vibration gray map, short-time Fourier transform time-frequency map, and continuous wavelet transform time-frequency map on the accuracy of diagnosis model are compared and analyzed. A very accurate guarantee is received, close to 100%. The final experimental results demonstrate the effectiveness of the information on the accuracy of diagnostic testing and provide new ideas for the verification and testing of wind turbine wind energy. Compared with other machine learning algorithms, the real-time recognition of machine learning based on time-domain statistical features is lower than that of convolutional neural network methods. The effect of the scale of the trained model on the accuracy of the algorithm is discussed. A sample ratio of 50% and 70% was found to be appropriate.

## 1. Introduction

As the main force of renewable energy, wind energy has also developed rapidly in recent years, and wind power generation and supporting technology are becoming more and more mature [1]. In addition, because the wind distribution factors need to be considered in the site selection of wind turbines, they are generally arranged in sparsely populated areas with remote geographical location and abundant wind resources. The influence of harsh working environment and weather factors will accelerate the aging speed of wind turbines, resulting in higher failure rate, lower service life, and higher operation and maintenance cost of wind turbines [2]. Although the capacity of wind turbines, the scale of wind turbines and the supporting force of technological progress are increasing year by year, and the performance and maintenance information of wind turbine operation monitoring and diagnosis are not suitable for its rapid development. This leads directly to timing errors and inaccuracies and maintenance of fans, which at least result in a financial loss of the wind farm, or a significant safety and security risk [3].

Rotating machinery is a kind of equipment widely used in modern industry. With the development of science and technology, rotating machinery and equipment are also developing in the direction of large-scale, sophisticated, and complex. For the rotating machinery and equipment of wind turbine, the monitoring of its state is mainly realized by means of signal analysis, including the analysis of the signals corresponding to the vibration, pressure, oil temperature, and other state quantities generated during the operation of the rotating mechanical equipment. The rotating parts on the transmission chain of wind turbine mainly include the rotor, bearing, and gearbox. However, poor working conditions in actual operation will lead to its failure. At present, the maintenance mode of wind turbine is mainly preventive maintenance, which itself has a certain lag. Wind power affects the local climate to some extent because it consumes wind power, which is an important factor in climate change. As a result, many scientists have focused on the destruction of wind turbines' early intelligence to facilitate improvements in failure and maintenance. Wind farms are serviced by many professional and efficient personnel and maintenance personnel, reducing the failure rate and maintenance cost of wind turbines [4].

At present, the fault diagnosis technology of wind turbine rotating parts uses expert experience for fault identification; that is, the fault characteristics of wind turbine vibration signal obtained by signal processing are manually identified and the diagnosis opinions are given, and the expert diagnosis process is shown in Figure 1. However, the diagnosis accuracy of this equipment diagnosis strategy depends on the diagnosis experience of experts, which will also lead to the rise of diagnosis cost and the diagnostic accuracy.

## 2. Literature Review

Sun et al. said that the current wind turbine fault diagnosis technology includes a signal processing-based method, model-based method, and data-driven method [5]. Gebraeel and Lawley adopt the automatic encoder (AE) network of five-layer network to realize the bearing fault diagnosis of motor. The model has the ability of self-adaptive fault feature extraction, and the classification accuracy is much higher than that of ordinary BP network [6]. Dong constructed a four-layer stacked sparse automatic encoder (SSAE) model. First, nonlinear projection compression was carried out on the input data, and adaptive feature extraction was carried out on the compressed one-dimensional data. The fault diagnosis of motor was realized. The classification accuracy reached 97.47%, which was much higher than the traditional shallow learning algorithm [7]. Shi et al. proposed a new method of rolling bearing fault diagnosis based on a convolutional neural network. Because CNN is suitable for image classification, the model first converts a one-dimensional signal into a two-dimensional image, which can achieve 100% accuracy by using the bearing data set of Case Western Reserve University in the United States. It also has strong robustness and antinoise ability [8]. Petrov et al. combine the historical data of wind turbine collected by the SCADA system with real-time data [9]. Urazghildiiev et al. completed the research on the life evaluation of wind turbine by combining artificial neural network and Bayesian algorithm and proved the effectiveness of the model by experiments [10]. Li et al. used hidden semi-Markov models (HSMM) to realize fault early warning of wind turbine and proposed a new method for training HSMM [11]. Jiang et al. estimate the model parameters through the improved forward-backward training algorithm, and its accuracy reaches 96% [12], which provides a theoretical and practical basis for Li et al.'s subsequent research [13]. Aiming at the problem of bearing fault diagnosis of wind turbine, combined with the analysis and processing of vibration signal and the in-depth learning method widely concerned and studied at present, especially the convolution neural network model technology, this study carries out feature learning and fault recognition of common bearing faults. The fault diagnosis method using vibration signal and convolution neural network model is studied, including signal processing, model design, model training, and model testing. First, various methods of converting the one-dimensional time-domain vibration signal into the two-dimensional image are analyzed, and the converted two-dimensional image is divided into the training set and test set. The training process is then sent to the convolutional neural network design of the research model, and the testing process is used to measure the diagnostic ability of the model. In addition, the number of layers and filters of the convolutional neural network and the training scale of the whole model are investigated.

## 3. Method

### 3.1. Fault Analysis of Wind Turbine Bearing

The rolling stones have been studied. A rolling mill usually consists of an inner ring, an outer ring, a rolling stock, and a cage, and this is the main basis of the bearing. Our three points are usually the result of damage and failure due to friction between the rolling surfaces of the rolling material and the inner and outer rings. Therefore, bearing failures usually occur on the inner ring, outer ring, and rolling elements. There are many reasons for failure. In addition to the deviation and other factors in the process of manufacturing and installation, the bad working environment and complex and changeable operating conditions will cause different forms and degrees of damage to the bearing [14]. At the same time, because the bearing has its own service life limit, long-term work itself will also lead to the degradation of the bearing. The common failure forms of bearing components mainly include fatigue, wear, fracture, corrosion, and deformation. Poor wear and lubrication, external dust particles and other foreign body invasions, improper transfer, and other reasons will aggravate the wear between the surface of the rolling bearing. When the degree of wear is serious, the bearing swimming gap increases and the surface roughness increases, which not only reduces the operation accuracy of the bearing, but also increases the vibration and noise of the equipment.

In the case of bearing failure, the recollision of the damage point with other material surfaces will focus on timely failure. These vibration disturbances are hallmarks of low vibration, and their specific frequency responses indicate local characteristics, with larger faults having greater effects [15]. The standard calculation method of the fracture frequency characteristic of each rolling bearing is as follows:

Inner ring fault frequency is calculated as follows:

(1) $$\begin{array}{c} f_{i}=\frac{N}{2}\left(1+\frac{d_{b}}{D}\cos\;\alpha \right)f_{r}. \end{array}$$

Outer ring fault frequency is calculated as follows:

(2) $$\begin{array}{c} f_{o}=\frac{N}{2}\left(1-\frac{d_{b}}{D}\cos\;\alpha \right)f_{r}. \end{array}$$

Rolling element failure frequency is calculated as follows:

(3) $$\begin{array}{c} f_{b}=\frac{N}{d_{b}}\left(1-{\left(\frac{d_{b}}{D}\cos\;\alpha \right)}^{2}\right)f_{r}. \end{array}$$

Cage failure frequency is calculated as follows:

(4) $$\begin{array}{c} f_{t}=\frac{1}{2}\left(1-\frac{d_{b}}{D}\cos\;\alpha \right)f_{r}. \end{array}$$

In the above formulas, *N* is the number of rolling elements, *D* is the diameter of the bearing, *d*_*b*_ is the diameter of the rolling elements, *α* is the contact angle, and *f*_*r*_ is the rotational frequency of the shaft. When a certain kind of fault occurs, the spectral peak of the corresponding fault frequency will appear in the bearing vibration spectrum. Considering the error of production, processing, installation, elastic deformation caused by load, interference of signal noise, and other factors, the actually observed fault frequency components may not be completely consistent with the formula calculation, but they are basically near the theoretical calculation value. Ideally, the fault type can be preliminarily judged based on this.

In addition, after being affected by the fault, the impulse shock may also cause high vibration of the bearing, and its vibration frequency is the natural vibration frequency of the bearing. In general, the natural frequencies of inner and outer bearings can reach several thousand Hertz, while the natural frequencies of rolling materials can reach several hundreds of Hertz. In natural vibration, the vibration performance of the inner and outer rings is the most obvious. The internal and external natural frequencies are shown in the following equation:

(5) $$\begin{array}{c} f_{n}=\frac{n\left(n^{2}-1\right)}{2\pi {\left(D/2\right)}^{2}\sqrt{n^{2}+1}}\sqrt{\frac{EI}{M}}. \end{array}$$

In the formula, *n* is the deformation coefficient, *E* is the elastic modulus of the material, the unit is 2 kg/m^2^, I is the inertia time of the ferrule section, *D* is the straight line intersecting the central axis, and *M* is the size of the long element. For the steel ball, its frequency can be expressed by formula (6), where *d* is the diameter and the material density:

(6) $$\begin{array}{c} f_{bn}=\frac{0.848}{\text{d}}\sqrt{\frac{E}{2\rho }}. \end{array}$$

### 3.2. Wind Turbine Vibration Signal Processing and Fault Diagnosis Method

At present, the operation process of mechanical vibration signal is generally divided into monitoring time, frequency analysis, and frequency measurement [16].

#### 3.2.1. Time Domain Analysis

Several indexes are counted according to the time-domain characteristics, and the dimensional parameters such as the value of dimensional parameters, absolute value, high value, square principle value, and square amplitude principle are diagnosed and tested. Dimensionless parameters, such as peak index, margin index, impact index, skewness index, and kurtosis index, should also be considered. Screening time is simple and intuitive, but uninterrupted data are limited. There are many problems with noise interference and complex fault signal processing. Due to the influence of the external harsh environment, fan rotating equipment is prone to failure and cause equipment vibration, and usually equipment vibration signal has strong nonstability and nonlinearity, so that the signal analysis of the fault features in the complex vibration signal extraction is the key step to realize the fault diagnosis.

#### 3.2.2. Frequency Domain Analysis

Frequency analysis typically includes magnitude spectrum, energy spectrum, energy spectrum, cepstrum, higher-order spectrum, and envelope spectrum. The magnitude spectrum is the distribution of magnitude over different frequencies. The energy spectrum, also known as the energy spectral density, is the signal strength within a frequency band. The energy spectrum is the signal strength within a unit frequency band and represents the variation of signal strength with frequency. The envelope spectrum can eliminate unnecessary frequency interference and highlight the fault characteristic frequency by taking the envelope signal for FFT after the Hilbert transform. It is mostly used to find early faults [17]. Frequency domain analysis can obtain rich and effective characteristic information to realize fault identification, but it is limited to stationary signal analysis [18].

#### 3.2.3. Time-Frequency Domain Analysis

Wind turbines are complex and have flexible operating conditions. Both record time analysis and test frequency can only delete one record data at a time, while analysis time takes into account the recorded time domain and frequency domain characteristic data, which is beneficial to nonstationary signal analysis. Frequency analysis time typically includes short-term Fourier transform (STFT), wavelet packet transform (WPT), Hilbert–Huang transform (HHT), S-transform, and Wigner–Ville distribution (WVD). It can convert a one-dimensional signal into a two-dimensional image signal with a time and frequency relationship. Time-frequency imaging constructed by combining texture features such as gray histogram and gray phase class matrix can be used for classification and recognition [19]. Adaptive nonstationary signal time-frequency analysis methods such as local mean decomposition (LMD) and empirical decomposition (EMD) are also widely used in fan gear and bearing fault detection.

In recent years, intelligent diagnostic programs have attracted extensive attention in the field of diagnosis. The essence of intelligent fault diagnosis is pattern recognition. Intelligent fault diagnosis is the product of the combination of artificial intelligence and fault diagnosis, which is mainly reflected in the field expert knowledge and the application of artificial intelligence technology in the diagnosis process. It is a system composed of people (especially field experts), hardware that can simulate brain function and its necessary external devices, physical devices, and software that supports these hardware. Regular and multifault states can be considered special models that can be ruled out and confirmed when extracting results. Among intelligent diagnostic procedures, critical point analysis (PCA) and independent analysis (ICA) are commonly used for specialty selection. Some classifications can select features during training, such as decision trees (DTs). Currently, classification based on statistical research procedures is most commonly used for intelligent diagnosis, including the KNN algorithm, random forest (RF) algorithm, support vector technology (SVM), and neural network device (ANN). With the rapid development of computer network technology and the integration of disciplines, mechanical and electrical equipment fault diagnosis technology moved from the original manual diagnosis to signal acquisition and analysis as the core of the remote intelligent monitoring and diagnosis of computers, such as CMS system, and moves in the direction of intelligent development.

Due to its automatic learning, in-depth research also provides new solutions for diagnosis. Deep learning standards are deep neural networks with many hidden processes that have a stronger negative impact on learning and crime research capabilities than standard learning systems. Common ones are deep reliability networks (DBNs), sparse autoencoders (SAEs), sparse filtering, convolutional neural networks, and recurrent neural networks (RNNs) [20, 21].

### 3.3. Convolutional Neural Network Theory

A typical convolutional neural network is usually composed of input layer, convolution layer, pooling layer, whole connection layer, output layer, and so on.  Figure 2 shows the model diagram of LeNet-5 network. Another design concept is also a combination of these network processes. The convolution pooling layer is the key to the strong image perception ability of the convolutional neural network, and it has the characteristics of sparse joints and heavy joints. The input is an image, including a one-channel grayscale image and three-channel color image. The output layer is generally a softmax classifier to output image classification and recognition results. For the field of target detection or image segmentation, there is a special output layer structure. The convolution layer is mainly used for feature learning, the pooling layer is used for feature selection, and the classifier uses the learned deep features for classification output. The network parameters of each layer are optimized at the same time in training [22]. The following sections focus on convolutional layers, pooling layers, fully connected layers, and classifiers.

After the convolutional neural network structure is designed, the depth of the network and the size and number of convolution kernels are determined, and the distribution is also known, but special connections (such as weights and unfairness) need to be studied and optimized. At the same time, the setting of training parameters such as learning rate is also very important. The unreasonable setting of training parameters may lead to overfitting or underfitting of model training and insufficient generalization ability of model. This section mainly introduces the basic objective function design and model training means [23].

The training of convolutional neural network can be regarded as an optimization problem, which needs to design an objective function to maximize or minimize the optimization goal. In the deep learning task, the cost function supplemented by the necessary regularization term is often used as the objective function. The cost function is a measure of the error between the classification prediction result and the actual truth value. The cost function commonly used in the classification task is the average value of the cross-entropy loss function of each sample. Cross entropy is a means to measure the similarity between two probability distributions. The target distribution is expressed as *p*(*x*) and the distribution obtained by prediction and estimation is expressed as *q*(*x*). The cross entropy between them is defined as follows:

(7) $$\begin{array}{c} H\left(p,q\right)=-\sum_{x}p\left(x\right)\log\;q\left(x\right). \end{array}$$

If the label value is represented by a one-hot vector, that is, the label value for *k* category classification is represented as the target vector with length k: [*p*^1^,…, *p*^*j*^,…, *p*^*k*^], if the target category is *y*_*i*_ = *c*, then *p*^*c*^ = 1 and other items are 0, and then the final objective function can be expressed as formula (8), where the expression 1{*c* = *yi*} indicates that if the condition in parentheses is true, then take 1; otherwise, it is 0.

(8) $$\begin{array}{c} L=-\frac{1}{m}\sum_{i=1}^{m}\sum_{c=1}^{k}1\left\{c=yi\right\}\cdot \;\log\frac{e^{z_{c}}}{\sum_{j=1}^{k}e^{z_{j}}}. \end{array}$$

### 3.4. Design of Wind Turbine Bearing Fault Diagnosis Algorithm Based on CNN

#### 3.4.1. Fault Diagnosis Process Based on CNN

Professional crime diagnosis often includes data acquisition, deletion, classification, etc. Rolling bearing is one of the most widely used rotating parts in mechanical equipment and is also one of the most easily damaged parts in mechanical equipment, and its good operation state will directly affect the performance of the whole machine, in which feature extraction is the key. Diagnosis neural networks based on the convolutional neural networks (CNNs) can transform diagnosis problems into similar images and partition tasks with the help of the energy function of automatically isolated features of deep learning models. Since the primary vibration signal is one dimensional, it must be specialized and converted into two-dimensional data before it can be transmitted to a two-dimensional convolutional neural network. In the experiments, the preliminary data are divided into training and experimental procedures. The training process is used to train the model, and the testing process is used to measure the capabilities of the model. In addition, the design and configuration of ultratrivial systems also need to be improved through experimentation and debugging.  Figure 3 shows the diagnosis process from sample acquisition to data preprocessing and then to model training. Once the model is trained and optimized, it can be used for the classification and identification of unknown state samples to diagnose whether the bearing state is healthy or not.

#### 3.4.2. Data Preprocessing

The original vibration data are a one-dimensional signal, which cannot be used for two-dimensional image recognition, so the data need to be converted.  Figure 4(a) shows the vibration data. The one-dimensional signal sampling values are rearranged into a two-dimensional matrix in order to make the vibration image (VI). Due to the limited original measurement data, overlapping sampling is carried out according to a certain length to increase the number of samples, as shown in Figure 4(b).

In this study, the length of a single signal sample (i.e. the number of sampling points contained in a single sample) is adjusted according to the actual sampling frequency and system rotation frequency. In order to facilitate convolution neural network processing, when the side length of the input image is an even number and the side length is an exponential power based on 2, it is more conducive to simplify the design of network structure parameters. The commonly used sample length is 400 = 20 × 20, 1024 = 32 × 32, 4096 = 64 × 64, etc.

In this study, short-term Fourier transform (STFT) and continuous wavelet transform (CWT) are also used as signal paths. The Fourier time shift represents the signal properties of the time signal past the time signal. The window length determines the time resolution and frequency resolution of the spectrum. The longer the window length, the longer the intercepted signal, the higher the frequency resolution after transformation, and the worse the time resolution. Fourier transforms a lot of functions and windows in a short period of time, and then Fourier transforms. The effects of Fourier switching are obtained by sliding window operations, and these effects are combined into a two-dimensional frequency table. The relevant formula is shown in equation (9), where *x*(*t*) represents the signal and *w*(*t*－*τ*) represents the window function. It can be seen that the short-time Fourier spectrum is a function of frequency *ω* and time *τ*:

(9) $$\begin{array}{c} X\left(\omega ,\tau \right)=<x\left(t\right),w\left(t－\tau \right)e^{j\omega t}>=\int x\left(t\right)\cdot w\left(t－\tau \right)e^{-j\omega t}\text{d}t. \end{array}$$

Since the large window of the short-time Fourier switch is fixed, it is only suitable for stable characters with small frequency fluctuations. The wavelet switch can adjust the window size according to the frequency and can bring out a variety of solutions. The definition of continuous wavelet transform is shown in equation (11), where equation (10) is wavelet basis function, and *s* and *τ* are scale factor and translation factor respectively, which respectively control the center frequency of wavelet transform and its translation along the signal on the time axis. Both *s* and *τ* take continuous variation values, which is a set of function series obtained from the same generating function *φ*(*t*) through expansion and translation. Therefore, the continuous wavelet transform is named. Because wavelet has two variables such as scale and translation, it can project the time signal onto the two-dimensional time-scale phase plane, which is conducive to extracting the characteristics of some time functions:

(10) $$\begin{array}{c} \varphi_{s,\tau }\left(t\right)=\frac{1}{\sqrt{s}}\varphi \left(\frac{t－\tau }{s}\right), \end{array}$$

(11) $$\begin{array}{c} W\left(s,\tau \right)=<x\left(t\right),\varphi_{s,\tau }\left(t\right)>=\frac{1}{\sqrt{s}}\int x\left(t\right)\cdot \varphi \left(\frac{t－\tau }{s}\right)\text{d}t. \end{array}$$

It can be seen from the above that compared with the grayscale image of the vibration signal, although the short Fourier transform and the continuous wavelet transform are complex, they have the advantage of solving some problems. This study makes an experimental comparative study on the above methods and then makes a trade-off between the effect of fault diagnosis and the complexity of analysis and processing.

#### 3.4.3. Model Design

In view of the similar structure of LeNet-5 convolutional neural network, this study preliminarily designs a network structure with three convolution pooling pairs and two full connection layers.

As the detection rate changes, the number of neurons in the urinary tract may increase if the types of violations increase, while the pattern of resection procedures continues to remain the same, so the network structure has some usability. In this study, the convolutional layer adopts the same filling method to keep the input and output size unchanged, and the pooling layer adopts an effective filling method, that is, no filling, so as to know the downsampling.  Table 1 lists the structural details of the convolutional neural network model, in which 32 × 32@16 means there are 16 channels, and the size of each channel is 32 × 32. Other items have similar meanings. The details and skills used for training include batch normalization and dropout. The convolutional layer and the fully connected layer use catch normalization to speed up the training, and the fully connected layer uses random deactivation to prevent overfitting of the structure and improve the generalization ability of the model. A recommended value of 0.5 is used for random deactivation compared in this table.

### 3.5. Experimental Verification and Example Analysis

To determine the effectiveness of the plan, a tensorflow framework was used for deep training. All tests were performed on a PC configured with an Intel Core i5 CPU and Geforce GTX 940 M GPU. The actual data of disease type rolling bed analysis are selected for analysis and evaluation. The left side of the rolling bearing test bed is a 2 horsepower (HP) motor to provide power source, the middle is a torque transmission device, and the right side is a load motor, which is also a dynamometer. In the experiment, the acceleration sensor is installed above the motor shell at the fan end and drive end respectively. In some experiments, the sensor is also installed on the base, and the sampling frequency per second is 12 kHz or 48 kHz. The fault bearing is installed at the drive end or the fan end for testing respectively. The fault defects are made by the electric discharge machining method. According to the fault location, it is divided into the inner ring, outer ring, and collision ring. In this experiment, bearing data were always measured at the end of actuation, and a frequency mode of 12 kHz was selected for analysis. The bearings used were set with three fault diameters, 0.007 inches, 0.014 inches, and 0.021 inches, representing different fault diameters. The above droplets with various failures and sizes were inspected and collected in four sizes (0, 1, 2, and 3 hp).

The final drive failures of the experiment are listed in Table 2. The fault frequency is a variety of frequency bands, calculated from the above error frequency. The same type of bearing is used in each experiment, and the location and size of fault points are different. Only one fault type is set at a time.

## 4. Results and Analysis

### 4.1. Preparation of Experimental Data

Under the same fault size and no-fault position, the measured vibration data of the three fault types are the same. In this experiment, the vibration signals of three fault locations, three fault sizes, and no fault, a total of 10 states are selected for analysis. The data measured under different loads with the same fault location and fault size are the same category, which are the time domain waveforms under 10 states when the load is 0 HP. N represents the normal state, BF, OF and IF represent ball rolling fault, outer ring fault, and inner ring fault, respectively, and 07, 14, and 21 represent three fault sizes. The bearing vibration signals of different fault types and fault degrees are obviously different, especially the total amplitude of the signal is also different due to the existence of fault impact components. For example, under normal conditions, the amplitude of bearing vibration signal is small and stable without an obvious impact component. When rolling element fault occurs, there is the obvious impact component, and the amplitude is also different under different fault degrees. It can also be seen from Table 3 that the time-domain signals under some fault types have a certain similarity, which is difficult to distinguish with the naked eye without signal processing, such as 0.014-inch and 0.021-inch outer ring faults [24].

The experimental data set is listed in Table 3. Overlapping samples are taken from the original vibration data under four load states. There are 10 states with different fault locations and fault degrees. There are 400 training samples and 200 test samples under each state, with a total of 6000 samples. The number of samples obtained for each type under each load condition is 150, which is a more appropriate data set size after considering the length of a single sample, the overlap rate, and the total length of the original vibration signal data.

### 4.2. Comparison of Signal Processing Methods

Here, we compare the signal processing of vibration grayscale Image (VI), short Fourier transform (STFT), and continuous wavelet transform (CWT). A vibrating grayscale image can only be seen by modifying the signal content by, for example, a sensor. Since there are no working data, key features of the data can be stored to be removed by the neural network. The vibration grayscale images of 9 fault types with different fault positions and different fault degrees are obtained. The sample signal length is 1024 points, and the size of the converted vibration grayscale image is 32 × 32. After different types of vibration signals are converted into vibration gray images, the texture shows different characteristics.

In this form, the short-time Fourier switch uses the Hamming window function, the main window is set to 64, the overlap value is set to 34, then the vibration signal of length 1024 can be converted to 33 × 32 time-frequency image, and 32 × 32 time-frequency image can be obtained after a simple operation, which can be directly sent to the convolutional neural network to obtain three fault types under 0 load and 0.007-inch fault size and the time-frequency diagram under normal state. There are obvious differences between them. Since the signal sampling frequency is 12 kHz, the time-frequency diagram obtained directly by the short-time Fourier transform covers the frequency of 0–6 kHz.

This study uses Matlab 2014a software for continuous wavelet transform, using cmor1-3 wavelet root function. The time-frequency map after wavelet transform is different from the short-time Fourier transform, and the time-frequency points are different. Because the time-frequency map after continuous wavelet transform has a high time axis resolution, it cannot be directly sent to the convolutional neural network. In this study, the original wavelet time-frequency map is compressed into 32 × 32 based on cubic spline interpolation. The vibration signal still retains the most important image features under rolling element fault before and after compression.

This experiment tests the 10 states established above. According to the different programs of a vibration signal, three control groups can be set. The experimental results are given in Table 4, from which it can be seen that the image frequency processed by our method is transmitted to the convolutional neural network, and the truth can be confirmed to be close to 100%, which proves that the processing of the information in this table is appropriate and effective. of.

It can also be seen from the table that the more complex the signal processing mode, the shorter the time required for model training. It shows that the complex signal processing has preliminarily extracted the fault characteristics of vibration signals, and the time-frequency diagrams are well distinguished, which reduces the difficulty of feature extraction of convolutional neural network, so the model converges quickly and has high accuracy. The method based on vibration gray image has high accuracy, but the training time is relatively long; This method does not need expert experience and complex signal processing. It can be seen from the above that the bearing fault diagnosis method based on the convolutional neural network can achieve good results in tasks with good data quality. When there is no complex signal processing and lack of expert experience, the vibration gray map method can be used to realize efficient bearing fault diagnosis.

### 4.3. Comparison with Machine Learning Methods

On the basis of contrasting traditional machine learning techniques and in-depth research, multiple time-domain statistics are selected according to features and are employed by a support vector machine (SVM), K-nearest neighbor classifier (KNN), and artificial neural network (ANN). The test results are shown in Figure 5.

From the test results, it can be seen that the validation rate of the machine learning technique based on temporal registration features is lower than that of the convolutional neural network process in clinical trials of various violation types. This is why it can be difficult to comprehensively observe and isolate the characteristics of vibration signals in different states, which limits the ability of machine learning models to distinguish between different types of signals. It is worth noting that while the design characteristics are similar, the accuracy tests of the three different machine technologies are also very close. This further proves that the factor limiting the recognition ability of machine learning model is the feature construction link, and the selection and optimization of the model itself is relatively secondary.

### 4.4. Discussion on the Proportion of Training Samples

Figure 6 shows the comparison between the accuracy of the model and the training time when the proportion of the training set is from 10% to 90%. It can be seen from the observation that with the increase of the proportion of training samples, the test accuracy of the model also increases but soon tends to saturation. For example, when the proportion increases from 50% to 70%, the increase of accuracy is not obvious. The training time of the obvious model increases as the model is trained. It can be seen from the analysis of the results that the ratio of the number of training standards to the number of test standards selected in this study is 4000 : 2000, and the percentage of training in the total data set is 67%, between 50% and 70%, which is also a reasonable distribution [25].

## 5. Conclusion

Based on the mechanical fault diagnosis of wind turbine gearbox bearings, this study analyzes the intelligent fault diagnosis process framework based on the convolutional neural network, which can solve the problem of high probability of mechanical faults of wind turbine bearings. It can effectively solve the problem of high probability of mechanical failure of fan bearings, meet the needs of automatic fault detection and intelligent operation and maintenance of fans, make up for the lack of poor fault diagnosis accuracy, and improve its fault diagnosis accuracy and early fault identification capabilities. The design method and diagnosis algorithm of deep convolution neural network model with three pairs of convolution pooling layers and two full connection layers are proposed. On this basis, combined with a public data set of a rolling bearing test rig, experiments are carried out on a practical mechanical fault diagnosis method. At the same time, according to the deep research model, exposure tests were carried out on the time-frequency imaging of the influence of three different vibration signal transformations, vibration grayscale images, short Fourier transform time-frequency images, and continuous wavelet transition time. The experimental results show that the system scheme has not been tested and is feasible. Future work will improve error detection and continue to apply smart test applications based on an in-depth study of error detection in different components of the gearbox, such as energy.

## Figures and Tables

**Figure 1:** Fault diagnosis process of fan rotating parts.

**Figure 2:** Structure diagram of typical convolution network LeNet-5.

**Figure 3:** Bearing fault diagnosis process based on CNN.

**Figure 4:** Signal preprocessing. (a) Vibration data. (b) Overlapping sampling.

**Figure 5:** Comparison of results of machine learning and deep learning methods.

**Figure 6:** Accuracy and training time under different proportions of training samples.

**Table 1:** Structure design of convolutional neural network.

Number of layers	Name	Nuclear size	Quantity	Output size	Activation function
1	Input layer	—	1	32 × 32@1	—
2	Convolution layer 1	5 × 5@1	16	32 × 32@16	ReLU
3	Pool layer 1	2 × 2@16	—	16 × 16@16	—
4	Convolution layer 2	3 × 3@16	32	16 × 16@32	ReLU
5	Pool layer 2	2 × 2@32	—	8 × 8@32	—
6	Convolution layer 3	3 × 3@32	64	8 × 8@64	ReLU
7	Pool layer 3	2 × 2@64	—	4 × 4@32	—
8	Full connection layer 1	512	1	512 × 1	ReLU
9	Full connection layer 2	128	1	128 × 1	ReLU
10	Output layer	10	1	10 × 1	Softmax

**Table 2:** Bearing parameters.

Inner diameter (inch)	Outer diameter (inch)	Thickness (inch)	Ball diameter (inch)	Pitch diameter (inch)	Inner ring fault frequency (kHz)	Outer ring fault frequency (kHz)	Cage failure frequency (kHz)	Rolling element fault frequency (kHz)
0.9843	2.0472	0.5906	0.3126	1.537	5.4152	3.5848	0.39828	4.7135

**Table 3:** Bearing fault diagnosis data set.

Load	Fault location		Fault size (inch)		
0–3	Rolling element	0.007	400	200	0
		0.014	400	200	1
		0.021	400	200	2
	Outer ring	0.007	400	200	3
		0.014	400	200	4
		0.021	400	200	5
	Inner ring	0.007	400	200	6
		0.014	400	200	7
		0.021	400	200	8
	No fault	—	400	200	9

**Table 4:** Diagnosis results based on CNN.

Diagnostic method	VI + CNN	STFT + CNN	CWT + CNN
Accuracy (%)	99.78	99.55	99.85
Training time (s)	258.30	10	1

## Data Availability

The data used to support the findings of this study are available from the corresponding author upon request.
